RETRACTED

# The Value of Echocardiography Combined with NT-pro BNP Level in Assessment and Prognosis of Diastolic Heart Failure

**DOI:** 10.1155/2022/2102496

**Published:** 2022-02-04

**Authors:** Shaolei Chen, Yanli Zhou, Xia Wu, Shaojun Shi, Haiyan Wu, Peng Li

**Affiliations:** Department of Ultrasound Medicine, Sinopharm Dongfeng General Hospital, Hubei University of Medicine, Shiyan 442008, Hubei, China

## Abstract

**Background:**

To investigate the significance of echocardiography combined with N-terminal pro-B-type natriuretic peptide (NT-pro BNP) levels in the evaluation and prognosis of diastolic heart failure (DHF).

**Methods:**

Clinical data were collected from 168 patients with DHF. Serum levels of NT-pro BNP were first measured by ELISA. Meanwhile, the echocardiography was used to examine left ventricular end-diastolic diameter (LVEDD), left ventricular diameter (LVD), and other parameters. Multivariate logistic regression analysis was performed for variables in heart failure assessment grade or poor prognosis. Finally, the predictive ability for New York Heart Association (NYHA) class as well as prognosis was assessed by ROC curves.

**Results:**

NT-pro BNP was the overexpression in the serum of patients with DHF. And the degree of elevation was related to NYHA class, while NT-pro BNP levels were significantly higher in the P-MACE group than in the N-MACE group. According to the multivariate logistic regression analysis, the ratio of peak velocity of left atrial early diastolic blood flow to early diastolic peak velocity of mitral annulus (*E*/Ea) and serum NT-pro BNP level was risk factors for NYHA class and prognosis. However, LVEF, LVEDD, and flow propagation velocity (Vp) can be a benefit condition. In addition, ROC curve showed that echocardiography combined with NT-pro BNP content had higher accuracy in NYHA class and prognostic assessment of DHF than applied separately.

**Conclusions:**

The diagnosis of echocardiography combined with NT-pro BNP levels has the potential to distinguish the NYHA class in heart function of patients with DHF and determine the prognosis of patients.

## 1. Introduction

Chronic heart failure (CHF) is a clinical syndrome of ventricular filling dysfunction and ejection dysfunction which caused by the cardiac structural damage and functional disturbances due to the various factors. Cardiac blood supply in CHF patients cannot meet the metabolic needs of other organs of the body [1]. According to the results of epidemiological survey in 2017, the prevalence of CHF is about 3% in developed countries in Europe or the Americas, and the prevalence is significantly increasing [2]. The prevalence of CHF in China is approximately 2%, and up to 500,000 new CHF patients are diagnosed each year [3]. Clinically, CHF is mainly divided into two types: systolic heart failure (SHF) and diastolic heart failure (DHF). Among them, DHF is more common. Surveys have shown that the number of patients with DHF accounts for more than half of the number of patients with CHF [4]. According to the report, the signs and symptoms of SHF and DHF are very similar, but there are huge differences in pathogenesis, ventricular remodeling, and treatment between them. At present, the research on SHF has been well investigated but the diagnosis and treatment of DHF are still being explored.

RETRACTED

DHF is also called heart failure with preserved ejection fraction (HFPEF). Its pathogenesis is due to the increased myocardial stiffness and slowed diastolic velocity, resulting in ventricular relaxation dysfunction or ventricular stiffness increasing, ultimately leading to abnormal ventricular filling and insufficient returned blood volume [5]. Moreover, the diagnosis of DHF is more difficult than that of SHF, which easily misses the optimal timing of early treatment for patients with DHF, resulting in poor prognosis or increased risk of death in patients with DHF [6]. At present, Doppler echocardiography is mostly used to evaluate left ventricular diastolic function for the diagnostic methods of DHF, and the main indicators include mitral annular velocity (Ea) and mitral valve bleeding velocity (*E*/*A*) [7]. This method can clearly observe the cardiac structural function and judge the hemodynamics. Factors such as subject's left ventricular load, valve regurgitation, and tester operating level easily affect the results of echocardiography, and this leads to a decrease in accuracy. Therefore, a single test cannot produce an accurate diagnosis.

In recent years, N-terminal pro-B-type natriuretic peptide (NT-pro BNP) as an inactive brain-type natriuretic peptide (BNP) in ventricular cell analysis [8], it has shown a significant role in the diagnosis, severity grading, and prognosis prediction of SHF [9, 10]. It has been pointed out that the concentration of NT-pro BNP in the blood can accurately reflect the mechanical function status of the heart and can be used as a biomarker of heart failure [11]. However, there are few studies on the value of NT-pro BNP in the diagnosis of DHF. Therefore, in this study, we investigated the value of echocardiography combined with NT-pro BNP level detection for the assessment and prognosis of DHF by collecting relevant data from patients with DHF.

## 2. Methods

### 2.1. General Information

Collected 168 patients with DHF visited our hospital from January 2016 to March 2019. All the collected patients complied the European Society of Cardiology (ESC) diagnostic criteria for DHF in 2007. According to the New York Heart Association (NYHA) cardiac function classification criteria, patients with DHF were divided into three subgroups: mildly symptomatic patients (NYHA II), moderately symptomatic (NYHA III), and severely symptomatic (NYHA IV). According to whether they had adverse cardiovascular events (MACE) during 1-year follow-up, patients with DHF were divided into major adverse cardiovascular event (MACE) group (P-MACE) and no MACE group (N-MACE). The control group was composed of healthy volunteers with normal heart function and left ventricular ejection fraction (LVEF) ≥ 50% and without severe heart disease and clinical symptoms of heart failure in the same issue. All subjects volunteered to participate in this study and were informed and consented.

RETRACTED

### 2.2. Screening Criteria

Inclusion criteria are as follows: meet the ESC diagnostic criteria for DHF in 2007 [12], have typical signs and symptoms of heart failure, LVEF was normal or slightly decreased, presented left ventricular diastolic dysfunction, and objective evidence of cardiac structural or functional abnormality. Exclusion criteria are as follows: patients with congenital heart disease, serious arrhythmia, pulmonary hypertension, pulmonary heart disease, malignant tumor, heart valve disease, hypertrophic cardiomyopathy, restrictive cardiomyopathy, pericardial disease, etc., at the same time, have serious liver and renal dysfunction, serious infection and mental disorders.

### 2.3. Measured the Level of NT-pro BNP in Serum by ELISA

5 mL venous blood was collected from all subjects at fasting state and centrifuged at 3000 r/min for 10 min at 4°C. The supernatant was removed in a new centrifuge tube and stored at -80°C. The level of NT-pro BNP in serum was detected strictly according to the steps in the package insert of NT-pro BNP ELISA assay kit.

### 2.4. Echocardiography Examination

Use Philips IE Elite Color Doppler ultrasound diagnostic instrument with 2-4 MHz frequency probe. Transthoracic ultrasonography was performed with the patient in the left lateral decubitus position, and the probe was closely attached to the sternum and apical regions of the subject to obtain two-dimensional and color Doppler flow images of the left ventricular long and short axis, apical long axis, apical four-chamber, and two-chamber views.

They recorded the following parameters: (1) left ventricular end-diastolic diameter (LVEDD), left ventricular diameter (LVD), left atrial diameter (LAD), peak early diastolic blood flow velocity (*E* value), and interventricular septum thickness (IVS) were measured on the left ventricular long-axis view. (2) Left ventricular ejection fraction (LVEF), flow propagation velocity (Vp), peak early diastolic velocity of mitral annulus (Ea), and *E*/Ea value were measured in apical four-chamber view and two-chamber view.

RETRACTED

### 2.5. Statistical Analysis

The data were analyzed by *χ*^2^ test using SPSS 21.0 statistical software, and the measurement data were expressed as mean ± standard deviation (SD). Used multivariate logistic regression analysis analyzes potential risk factors for variables with statistically significant differences in heart failure assessment grades (NT-pro BNP, LVD, IVS, *E*/Ea, LVEF, LVEDD, Vp) and variables with statistically significant differences in prognosis (NT-pro BNP, IVS, *E*/Ea, LVEF, LVEDD, Vp). ROC curves were plotted to calculate the area under the curve (AUC) and judge the predictive ability of echocardiography and NT-pro BNP single or combined application for the poor prognosis of DHF. Differences were considered statistically significant at *P* < 0.05.

## 3. Results

### 3.1. Basic Information

The basic information of all subjects was shown in Supplementary Table 1. There were significant differences between the DHF group and the control group in terms of body mass index (BMI), history of diabetes and hypertension, total cholesterol (TC), high-density lipoprotein (HDL), and low-density lipoprotein (LDL) levels (*P* < 0.05). However, there were no significant differences in age, gender, smoking history, and triglyceride (TG) levels between the two groups (*P* > 0.05).

### 3.2. Serum NT-pro BNP Levels Are Elevated in Patients with DHF

The results of ELISA showed that the levels of serum NT-pro BNP in patients with DHF were significantly increased compared with the control group, and the higher levels of NYHA class, the NT-pro BNP level also increased (Figure 1(a)*P* < 0.05). This result illustrated that serum NT-pro BNP levels were significantly increased in patients with DHF, and that the more severe the DHF grade, the more significant the increase in NT-pro BNP levels. In addition, we divided the patients into the P-MACE group (*n* = 87) and N-MACE group (*n* = 81) according to whether MACE occurred. ELISA results showed that the serum NT-pro BNP level in the P-MACE group was significantly increased than that in the N-MACE group (Figure 1(b)*P* < 0.05).

### 3.3. Comparison of Echocardiographic Parameters

Echocardiography was used to further detect DHF related parameters in four sections of the heart in patients with DHF: long and short axis, apical long axis, apical four-chamber, and two-chamber sections (Figure 2). The results showed that compared with the control group, the values of LVD, IVS, and *E*/Ea were significantly increased in patients with DHF, while the values of LVEDD, LAD, LVEF, and Vp were significantly lower (Table 1, *P* < 0.05). Cardiac parameters were further compared across NYHA class in patients with DHF. It was found that the values of LVD, IVS, and *E*/Ea were significantly higher in the NYHA IV and NYHA III group than in the NYHA II group and higher in NYHA IV than in the NYHA III group. The values of LEVDD, LAD, LVEF, and Vp were significantly lower in the NYHA IV group compared with the NYHA II group (Table 1).

RETRACTED

### 3.4. Basic Information of DHF Patients with or without Cardiovascular Events

As shown in Supplementary Table 2, there were significant differences between the two groups only in terms of age and history of hypertension. Other indicators such as gender, smoking history, and history of diabetes mellitus did not differ significantly between the two groups.

### 3.5. Relationship between whether MACE Occur and Echocardiographic Parameters in Patients with DHF

We then compared the differences in cardiac parameters between patients in the N-MACE and P-MACE groups. As shown in Table 2, patients in the P-MACE group had significantly higher IVS and *E*/Ea values and significantly lower LEVDD, LVEF, and Vp values compared with the N-MACE group (Table 2, *P* < 0.05), while the differences in LVD and LAD values between the two groups were not statistically significant (*P* > 0.05).

### 3.6. Multivariate Logistic Regression Analysis

#### 3.6.1. Factors Influencing DHF Grading

Multivariate logistic regression analysis of the variables with statistically significant differences in heart failure assessment showed that *E*/Ea and the level of NT-pro BNP serum could be risk factors for NYHA class. LVEF, LVEDD, and Vp could be favorable factors for NYHA class (Tables 3 and 4).

#### 3.6.2. The Prognostic Factors of DHF

Multivariate logistic regression analysis was performed on variables with statistically significant prognosis. The results showed that *E*/Ea and NT-pro BNP were risk factors for MACE in patients, and LVEF, LVEDD, and Vp were protective factors for MACE in patients (Table 5, *P* < 0.05).

### 3.7. The Role of Echocardiography and NT-pro BNP in the Evaluation and Prognosis of Patients with DHF

The diagnostic value of echocardiography and NT-pro BNP levels for NYHA class or prognosis was assessed by the ROC curve analysis. Echocardiography combined with NT-pro BNP had higher accuracy in identifying NYHA III (AUC: 0.771) and NYHA IV (AUC: 0.985) than echocardiography or NT-pro BNP level assessment alone (Figures 3(a) and 3(b) and Table 6). In addition, in terms of the potential predictive value of the prognosis of DHF, echocardiography combined with NT-pro BNP level (AUC: 0.904) also had higher accuracy than those of echocardiography and NT-pro BNP level used independently (Figure 3(c) and Table 6).

RETRACTED

## 4. Discussion

BNP and NT-pro BNP are significance in the diagnosis of heart failure, and they also have auxiliary value in evaluating the severity and prognosis of heart failure. NT-pro BNP is decomposed from BNP released by myocardial cells. It has the characteristics of stable chemical structure, small difference among individuals, and long half-life which has more clinical value than BNP. Nowadays, NT-pro BNP plays an important role in the diagnosis, classification, and treatment of chronic heart failure, and some studies have applied it to the prognosis of heart failure [13]. Some studies have shown that the blood concentration of NT-pro BNP in patients with DHF is increased [14]. And other studies have shown that the level of NT-pro BNP can predict the risk of adverse cardiovascular disease [15]. In this paper, ELISA results showed that serum NT-pro BNP levels in patients with DHF were significantly increased; with the increase of the severity of grading, the degree of increase is more significant, compared with DHF patients without mace, and the serum NT-pro BNP level of DHF patients with poor prognosis was higher. At the same time, this study through multivariate logistic regression analysis found that NT-pro BNP was a risk factor for MACE and NYHA class in patients, which means that NT-pro BNP is can be the basis for grading and prognosis of patients with DHF. However, there are some studies have shown that men have lower NT-pro BNP levels than women [16]. Renal dysfunction leads to sodium-water retention, resulting in increased cardiac pressure load, and finally increased left ventricular wall pressure, resulting NT-pro BNP release [17]. This suggests that the level of NT-pro BNP in blood may be affected by gender or renal function. Therefore, use of the single NT-pro BNP method is not comprehensive for the grading diagnosis and prognosis of DHF, and other diagnostic methods are needed.

Among them, the main judgment indexes of DHF determined by Doppler ultrasound include *E*/Ea > 8, LVEDP > 15 mmHg, and LVEF > 50%. The results of other studies showed that the decrease of LVEDD, Vp, and LVEF was the factor of DHF produced [18, 19]. Other studies have shown that Vp < 45 cm/s is the left ventricular diastolic dysfunction [20]. The results of this study showed that compared with the control group, the LVD, IVS, and *E*/Ea values of DHF patients were significantly increased, and the LVEF, LAD, LVEDD, and *Vp* values were significantly decreased. At the same time, compared with the N-MACE group, IVS and *E*/Ea in the P-MACE group were significantly increased, while LVEF, LVEDD, and Vp were significantly decreased. These results indicate that echocardiography can evaluate the classification and prognosis of DHF through *E*/Ea, LVEDP, LVEF, and other indicators, but there was no statistical significance of difference in IVS, LVEF, and LVEDD between NYHA III and NYHA IV subgroups, indicating that echocardiography cannot clarify the standard difference between NYHA III and NYHA IV. Through multiple factor logistic regression analysis, further found that *E*/Ea is a risk factor for NYHA class and MACE in DHF patients, while LVEF, LVEDD, and Vp are favorable factors. Although previous studies have shown that *E*/Ea value is the gold standard for DHF evaluation and prognosis judgment [21], it is difficult to accurately calculate the ratio of *E*/Ea due to the measurement of *E* and Ea in different cycles and different load states and the instability of *E* and Ea in DHF patients; moreover, the measurement repeatability of LVEDD, Vp, and LVEF is poor, which is not conducive to clinical development. Therefore, this study considered use echocardiography combined with NT-pro BNP level to evaluate DHF and prognosis.

RETRACTED

With the development of recombinant protein technology, in clinic, the detection results of NT-pro BNP are more stable and reliable, and the operation of NT-pro BNP is more convenient, which can avoid the deviation of echocardiography caused by different operation. At the same time, the detection results of NT-pro BNP can make up for the shortcomings of echocardiography, such as the unclear standard difference between NYHA III and NYHA IV. Echocardiography can provide the information of cardiac cavity size and wall thickness, which can avoid the deviation of NT-pro BNP content as the standard caused by gender or renal function. Therefore, in clinical practice, echocardiography and NT-pro BNP are often used in combination to diagnose diseases. The research shows that echocardiography combined with NT-pro BNP can be used to diagnose percutaneous transvenous mitral commissurotomy [22], subclinical cardiotoxic [23], heart failure [24], and other diseases. Therefore, this study explored the effect of echocardiography combined with NT-pro BNP detection on DHF grading evaluation and prognosis. The results showed that echocardiography combined with NT-pro BNP content had higher accuracy in NYHA class and prognostic assessment of DHF than those of echocardiography and NT-pro BNP separate application.

## 5. Conclusion

In conclusion, echocardiography combined with NT-pro BNP level has the potential to distinguish the NYHA class of DHF patients and judge the prognosis of DHF patients. However, in this study, the cases collected by a single medical institution are limited in region and number of cases, which cannot fully represent all DHF patients. Therefore, it is still need a further research to better illustrate the diagnostic value of echocardiography combined with NT-pro BNP.

RETRACTED

## Figures and Tables

**Figure 1:** Serum NT-pro BNP levels in patients. (a) Serum NT-pro BNP levels are elevated in patients with DHF. (b) Increased serum NT-pro BNP level in patients with DHF in the P-MACE group. ∗∗∗*P* < 0.001.

**Figure 2:** Echocardiography of patients with DHF.

**Figure 3:** The role of echocardiography and NT-pro BNP in the evaluation and prognosis of patients with DHF. (a) ROC curve analysis of NYHA III diagnosis. (b) ROC curve analysis of NYHA IV diagnosis. (c) ROC curve analysis of MACE diagnosis in patients.

**Table 1:** Echocardiographic measures were compared between the control group and each NYHA class group of DHF.

Characteristics	Control (*n* = 60)	DHF (*n* = 168)			
		Total (*n* = 168)	NYHA II (*n* = 51)	NYHA III (*n* = 78)	NYHA IV (*n* = 39)
LVEDD (mm)	48.38 ± 2.32	42.77 ± 3.53^∗^	45.22 ± 2.96^∗^	42.09 ± 3.19^∗^^#^	40.92 ± 3.17^∗^^#&^
LVD (mm)	45.82 ± 0.76	51.72 ± 2.78^∗^	50.78 ± 1.73^∗^	51.64 ± 2.29^∗^^#^	53.12 ± 4.01^∗^^#&^
LAD (mm)	34.18 ± 3.15	31.69 ± 3.10^∗^	32.33 ± 3.18^∗^	31.45 ± 2.86^∗^	31.33 ± 3.38^∗^
IVS (mm)	8.96 ± 1.22	10.78 ± 0.87^∗^	10.03 ± 0.60^∗^	10.94 ± 0.74^∗^^#^	11.45 ± 0.70^∗^^#&^
LVEF (%)	60.98 ± 2.82	53.99 ± 5.42^∗^	56.64 ± 5.30^∗^	54.59 ± 4.67^∗^^#^	49.34 ± 3.96^∗^^#&^
Vp (cm/s)	0.54 ± 0.02	0.490 ± 0.04^∗^	0.50 ± 0.04^∗^	0.49 ± 0.03^∗^	0.45 ± 0.04^∗^^#&^
*E*/Ea	6.16 ± 0.58	11.29 ± 1.54^∗^	9.49 ± 0.92^∗^	11.84 ± 0.86^∗^^#^	12.52 ± 1.12^∗^^#&^

Data were mean ± SD. ^∗^*P* < 0.05, compared with control; ^#^*P* < 0.05, compared with NYHA II; ^&^*P* < 0.05, compared with NYHA III. DHF: diastolic heart failure; NYHA: New York Heart Association; LVEDD: left ventricular end-diastolic diameter; LVD: left ventricular diameter; LAD: left atrial diameter; IVS: interventricular septum thickness; LVEF: left ventricular ejection fraction; Vp: flow propagation velocity; *E*/Ea: peak early diastolic blood flow velocity/peak early diastolic velocity of mitral annulus.

**Table 2:** Comparison of echocardiographic indicators in patients with DHF with cardiovascular events.

Characteristics	N-MACE (*n* = 81)	P-MACE (*n* = 87)	*P* value
LVEDD (mm)	44.56 ± 3.02	41.11 ± 3.15	<0.001
LVD (mm)	51.56 ± 2.27	51.87 ± 3.18	0.47
LAD (mm)	31.89 ± 3.26	31.49 ± 2.94	0.41
IVS (mm)	10.53 ± 0.85	11.02 ± 0.83	<0.001
LVEF (%)	56.62 ± 4.71	51.55 ± 4.89	<0.001
Vp (cm/s)	0.49 ± 0.04	0.48 ± 0.05	0.02
*E*/Ea	10.49 ± 1.31	12.02 ± 1.36	<0.001

Data were mean ± SD.

RETRACTED

**Table 3:** Multivariate logistic regression analysis of NYHA II and NYHA III.

Variables	Regression coefficient	Standard error	*Z* value	Wald *χ*^2^	*P* value	OR value	95% CI
NT-pro BNP	0.003	0.001	1.87	3.498	0.061	1.003	1.000~1.005
LVEF	0.118	0.09	1.305	1.702	0.192	1.125	0.943~1.342
Vp	15.879	12.83	1.238	1.532	0.216	7.87^10^6^	0.000~6.56×10^17^
*E*/Ea	3.197	0.777	4.114	16.923	≤0.001	24.45	5.332~112.125
LVD	0.25	0.224	1.117	1.248	0.264	1.284	0.828~1.993
IVS	1.319	0.695	1.899	3.607	0.058	3.74	0.959~14.592
LVEDD	-0.2	0.141	-1.421	2.02	0.155	0.819	0.621~1.079

**Table 4:** Multivariate logistic regression analysis of NYHA III and NYHA IV.

Variables	Regression coefficient	Standard error	*Z* value	Wald *χ*^2^	*P* value	OR value	95% CI
NT-pro BNP	0.009	0.002	4.269	18.225	≤0.001	1.009	1.005~ 1.014
LVEF	-0.146	0.117	-1.241	1.541	0.214	0.864	0.687~ 1.088
Vp	-8.283	15.617	-0.53	0.281	0.596	0.000	0.000~ 4.96×10^9^
*E*/Ea	2.842	0.837	3.397	11.541	0.001	17.153	3.328~ 88.407
LVD	0.303	0.252	1.201	1.442	0.23	1.353	0.826~ 2.218
IVS	2.526	0.877	2.879	8.291	0.004	12.505	2.240~ 69.800
LVEDD	0.067	0.177	0.381	0.146	0.703	1.07	0.757~ 1.512

**Table 5:** Multivariate logistic regression analysis of MACE Occurrence.

Variables	Regression coefficient	Standard error	*Z* value	Wald *χ*^2^	*P* value	OR value	95% CI
NT-pro BNP	0.002	0.001	2.216	4.911	0.027	1.002	1.000~ 1.003
LVEF	-0.151	0.048	-3.155	9.955	0.002	0.86	0.783~ 0.944
Vp	6.631	5.786	1.146	1.314	0.252	758.397	0.009~ 6.378×10^7^
*E*/Ea	0.482	0.204	2.368	5.609	0.018	1.619	1.087~ 2.413
IVS	-0.382	0.295	-1.293	1.673	0.196	0.683	0.383~ 1.218
LVEDD	-0.214	0.071	-3.01	9.058	0.003	0.808	0.703~ 0.928

**Table 6:** Analysis of the ROC curves for the NYHA III, NYHA IV, and MACE-grade diagnoses.

	AUC	Sensitivity	Specificity
NYHA III			
NT-pro BNP	0.751	0.647	0.804
Echocardiography	0.584	0.255	1
Echocardiography combined with NT-pro BNP	0.771	0.98	0.431
NYHA IV			
NT-pro BNP	0.955	0.923	0.872
Echocardiography	0.876	0.718	0.897
Echocardiography combined with NT-pro BNP	0.985	1	0.897
MACE			
NT-pro BNP	0.758	0.483	0.914
Echocardiography	0.813	0.77	0.741
Echocardiography combined with NT-pro BNP	0.904	0.77	0.901

## Data Availability

The data used to support the findings of this study are available from the corresponding author upon request.

## Supplementary Materials

Supplementary 1 Supplementary Table 1: comparison of the general data of each NYHA class between the control group and DHF.

Supplementary 2 Supplementary Table 2: comparison of general data of DHF patients with or without cardiovascular events.
